The article "Entrepreneurial Willingness, Practice, and Management Path of College Graduates in a Green Development Environment" was published in 2022. Journal: J Environ Public Health.

# Entrepreneurial Willingness, Practice, and Management Path of College Graduates in a Green Development Environment

**DOI:** 10.1155/2022/5453097

**Published:** 2022-09-26

**Authors:** Fei Ma

**Affiliations:** School of Marxism, Henan Agricultural University, Zhengzhou, Henan 450046, China

## Abstract

Before entrepreneurial behavior occurs, individual personality traits have a very important impact on the formation of entrepreneurial willingness. The purpose of this research is to explore the entrepreneurial intention, practice, and management path of college graduates in a green development environment. In this study, three dimensions of green entrepreneurial traits (risk propensity, ecological values, and social responsibility) and three dimensions of green entrepreneurial motivation (fame and fortune motive, spiritual motive and responsibility motive, and green entrepreneurial intention) are determined, and a questionnaire is compiled. Then, the questionnaire survey data of college graduates is collected, and a structural equation model is constructed. The influence of risk tendency, ecological values, and social responsibility on green entrepreneurship motivation is studied in turn, and the influence of fame and fortune motive, spiritual motive, and responsibility motive on green entrepreneurship willingness is explored. Finally, the mediating role of the three dimensions of green entrepreneurial motivation in the influence of green entrepreneurial traits on green entrepreneurial willingness is tested. The study finds that the average score of families with entrepreneurial experience was 4.0526. The average score of families without entrepreneurial experience was 3.6463, and the significance index was at the level of 0.001. The same results as previous scholars have appeared, that is, students with entrepreneurial family background have stronger (green) entrepreneurial willingness. Green entrepreneurship creates green value through green products or services, drives green consumption, leads green values, and contributes to the sustainable development of society and ecology.

## 1. Introduction

In the current era of difficult employment for college students, although the state strongly supports innovation and entrepreneurship, the entrepreneurship rate of college students is still low. As an emerging entrepreneurial method, green entrepreneurship can not only solve the problem of college students' employment difficulties and stimulate economic growth, but also lead green consumption and spread green values, contributing to the sustainable development of the ecological environment. Understanding the structure and characteristics of college students' green entrepreneurial traits and green entrepreneurial motivation and deeply analyzing the impact and mechanism of the two on green entrepreneurial willingness of college students can help the education department identify potential green entrepreneurs. It is also possible to formulate clearer training goals and programs, encourage, and support more college students to invest in green entrepreneurship, so as to help more people put their green entrepreneurship will into practice. With the increasingly serious ecological and environmental problems, from environmental protection, sustainable development, ecological civilization, beautiful China to the concept of green development, it is the logical necessity of the continuous deepening of the ecological value proposition. The related research on college students as the object of education has also been deepened.

In the research on green entrepreneurship, there are very few researches on green entrepreneurship willingness by scholars, and few articles deal with the influence of personal characteristics on green entrepreneurship willingness. Radu-Lefebvre et al. argued that entrepreneurial legitimacy is described as a trigger for entrepreneurial career choice and motivation, which means that an individual's propensity to pursue an entrepreneurial career increases with the social legitimacy of the career [1]. Dutra's research data on entrepreneurial willingness was not very rich. He reviewed previous articles and optimized entrepreneurial willingness based on the green development environment. As one of the five development concepts related to the overall economic and social development, the concept of green development has a strategic, programmatic, and leading role [2]. Voda et al. believed that unemployment among young people has become a particularly serious problem [3]. Decreton et al. believed that the headquarters of multinational companies can help the development and transfer of innovative ideas of subsidiaries [4]. Ebrahimi and Mirbargkar assessed the role of green entrepreneurship [5]. Mrkajic et al. studied the selection bias between green and nongreen entrepreneurs [6]. Demirel et al. believed that the number of green start-ups is steadily increasing [7]. Yang et al. believed that green entrepreneurship is a special type of entrepreneurship that can achieve sustainable development and is advocated by many countries and regions [8]. Song and Lee believed that positive relationships are important for the skills and personal development required for entrepreneurship [9]. Green development is shared by everyone, and everyone is responsible. College students are the hope of the nation and the future of the motherland. The value orientation of green development will greatly affect the value orientation of the whole society in the future, and it is the key object of education on the concept of green development. The green development environment will be further introduced later.

This study takes college graduates as the object; explores the relationship between green entrepreneurial characteristics, green entrepreneurial motivation, and green entrepreneurial willingness of college graduates; and builds a theoretical model based on this. Combined with the existing research, the corresponding research hypotheses are put forward according to the theoretical model designed in this research. After confirming the scope and object of investigation, referring to the existing mature scales, and combining with the theoretical assumptions put forward, the initial questionnaire is drawn up. In the process of model validation, AMOS24 software is used to construct the structural equation model between variables. Firstly, the fit degree of the structural equation conceptual model is evaluated by using the model fit index. The survey of green entrepreneurial willingness finds that the standardized factor loadings of the five items of green entrepreneurial willingness are all greater than 0.5. Therefore, it is suitable for the next test of CR and AVE. The CR value obtained by calculation is 0.903, which is greater than 0.7. The AVE is 0.653, which is greater than 0.5. The results of ecological values study showed that the CR value was 0.840, which was greater than 0.7, and the AVE value was 0.568, which was greater than 0.5.

## 2. Method of Entrepreneurial Intention, Practice, and Management Path

### 2.1. Entrepreneurial Willingness

Willingness is an individual's subjective attitude toward a particular behavior. It helps predict actual behavior and reflects commitment to future actions. At the end of the twentieth century, under the dual role of market and ecological orientation, green entrepreneurship came into being. With the development of green entrepreneurship practice, the research on green entrepreneurship is also deepening, but scholars have no unified conclusion on the definition of green entrepreneurship so far. According to the theoretical analysis of entrepreneurial willingness and green entrepreneurship in this study, this research defines the green entrepreneurial willingness of college graduates as a subjective attitude of individual college graduates about whether to carry out green entrepreneurship in the future. This subjective attitude can predict whether they will conduct green entrepreneurship in the future. The influencing factors of entrepreneurial intention are shown in Figure 1. The measurement of entrepreneurial willingness can well identify potential entrepreneurs. Many scholars have done a lot of research on entrepreneurial willingness, but the research on green entrepreneurial willingness is relatively scarce. In addition, in the existing research, most of the influencing factors of entrepreneurial intention are from the personality traits of entrepreneurs, the external entrepreneurial environment and the entrepreneurial policies of the government or schools. Meanwhile, some studies have shown that entrepreneurial motivation is affected by the personal characteristics of entrepreneurs. However, existing research has not systematically considered the mediating role of entrepreneurial motivation in the relationship between entrepreneurial personality traits and entrepreneurial intention. Therefore, this paper explores potential green entrepreneurs by studying the relationship between green entrepreneurial characteristics, green entrepreneurial motivation, and green entrepreneurial willingness of college graduates. From the perspective of behavioral psychology, the prediction mechanism of individual psychology on behavior is discussed, specific green entrepreneurial situations are given, and psychological characteristics can more accurately predict which psychological characteristics can increase the possibility of their green entrepreneurial practice.

The independent variable *X* has an influence on the dependent variable *Y*, and *M* acts as an intermediary variable. *X* can influence *Y* through *M*. The relationship between variables can be described by the following regression equation as [10]

(1) $$\begin{array}{c} Y=cX+e_{1}, \end{array}$$

(2) $$\begin{array}{c} M=abX+e_{3}, \end{array}$$

(3) $$\begin{array}{c} Y_{2}=cX+\text{bm}+e_{3}. \end{array}$$

Among them, *c* represents the direct effect of *X* on *Y* after controlling for *M* [11].

The product of the elements of each row of the matrix is calculated as [12]

(4) $$\begin{array}{c} m_{i}=\prod a_{ij}. \end{array}$$

The *n*-th root of *m*_*i*_ is calculated as

(5) $$\begin{array}{c} W_{i}=\sqrt[{n}]{m_{i}.} \end{array}$$

It is normalized through [13]

(6) $$\begin{array}{c} w_{g}={\left(W1,W2,\cdots Wn\right)}^{T}. \end{array}$$

The largest eigenvalue *λ*max is computed as

(7) $$\begin{array}{c} \lambda \max=\frac{1}{N}\sum \frac{A}{W}. \end{array}$$

The index CI of the inconsistency of matrix *A* is calculated as [14]:

(8) $$\begin{array}{c} \text{CI}=\frac{\left[\partial \left(A\right)-n\right]}{\left(n-1\right)}. \end{array}$$

Green entrepreneurs focus on sustainable strategies, that is, emerging technologies, markets, suppliers, customers, and other stakeholders, which mean breakthrough innovation. Sustainability here includes two possible aspects. One aspect refers that green entrepreneurship is a structural system, and all elements and links in the system, including entrepreneurial motivation, process, and team spirit, should have a neutral or positive impact on the environment. The other is that some aspects of the entire green entrepreneurship process are in line with green requirements, while other aspects may not necessarily meet. The index CR of the consistency of matrix *A* is calculated as [15]

(9) $$\begin{array}{c} \text{CR}=\frac{\theta \text{CI}}{\text{RI}}. \end{array}$$

### 2.2. Green Development Environment

Willingness is the precondition of individual behavior, and entrepreneurial willingness under green development environment is the key link in entrepreneurial research under green development environment. Personality traits of individuals have an important impact on their entrepreneurial intentions. Entrepreneurship in a green development environment has higher requirements on the entrepreneur's personality traits such as risk inclination, ecological values, and social responsibility. The entrepreneurial theory believes that entrepreneurial motivation is an effective indicator to predict the entrepreneurial willingness and behavior of individuals. The main techniques of the study are shown in Figure 2. Different dimensions of motivation have different degrees of influence on the formation of entrepreneurial intention. Entrepreneurs in a green development environment may have the will to start a business in a green development environment out of motivations such as gaining fame and fortune, realizing spiritual pursuits, and taking on environmental protection and social responsibilities. Previous studies have found that personality traits such as risk-taking tendencies have an impact on entrepreneurial motivation. Entrepreneurial activities in a green development environment have higher risks, and individuals with strong ecological values and social responsibility are more likely to engage in entrepreneurial activities in a green development environment. Therefore, entrepreneurial motivation in a green development environment is likely to be affected by individual risk tendencies, ecological values, and social responsibility.

The arc elasticity coefficient *R* in economics is introduced as [16]

(10) $$\begin{array}{c} R=\frac{\left(N/M\right)}{\left[N/\left(M1+M2\right)\right]}. \end{array}$$

Green entrepreneurship stability is *Z*_*M*_, as shown in

(11) $$\begin{array}{c} \delta =\frac{\pi }{2\left(g+h+i+e+t\right)}. \end{array}$$

The diffusion efficiency of entrepreneurial behavior in the whole group of college graduates will be affected.

The essence of entrepreneurship is innovation and change, and innovative green business practices can bring competitiveness while improving environmental performance. Ecoentrepreneurship builds a bridge between business success and protection of the ecological environment through environmental innovation. The difference between their ecological entrepreneurship and other entrepreneurship is that they are oriented to protect the ecological environment, and most of this way of protecting the ecological environment is achieved through innovation. Influence coefficients *δ*_*J*_ and *δ*_*I*_ for diffusion between entrepreneurial behaviors can be obtained through

(12) $$\begin{array}{c} \delta_{J=}\delta_{I}\left(G,H,I,E,T\right), \end{array}$$

(13) $$\begin{array}{c} \delta_{I=}\delta_{CE}\left(G,H,I,E,T\right). \end{array}$$

Expression in mathematical mode: it is supposed that the input set of subject *M* is *Z*_*M*_ [17]:

(14) $$\begin{array}{c} Z_{M}=\left\{Z_{1},Z_{2},\cdots ,Z_{N}\right\}. \end{array}$$

The output set is *Y*_*M*_ [18]:

(15) $$\begin{array}{c} Y_{M}=\left\{Y_{1},Y_{2},\cdots ,Y_{N}\right\}. \end{array}$$

Since the input determines the output, there is

(16) $$\begin{array}{c} Y=F\left(XV\right). \end{array}$$

Compared with ordinary entrepreneurship, green entrepreneurship has higher requirements for product or service innovation, and the market entry threshold is higher. Meanwhile, the awareness of green consumption among Chinese residents is not strong enough, so green entrepreneurship is more difficult to succeed than ordinary entrepreneurship. Although people with high-risk propensity are willing to experience high-risk entrepreneurial activities, relatively speaking, their ecological environment protection concept and social responsibility have a greater role in promoting the formation of their green entrepreneurial willingness. Gray evaluation weight Re of the *e*-th gray category of evaluation index *V* is shown as

(17) Re=XiXj.

Then, the gray evaluation weight vector of each gray category is obtained as [19]

(18) $$\begin{array}{c} r_{11}=\left[m\right]\left(\begin{array}{ccc} r_{1} & \cdots & r_{151}\\ \vdots & \ddots & \vdots \\ s_{11} & \cdots & s_{11} \end{array}\right). \end{array}$$

Comprehensive evaluation of the awareness of college graduates' self-employment support system is

(19) $$\begin{array}{c} G=\text{HQ}=\left[H_{1}\cdots H_{N}\right]. \end{array}$$

If the adoption of implementation behavior *a* (entrepreneurial behavior) leads to different profit and loss values *w*, the probability of being finally realized is *P*. If the implementation behavior *b* (nonentrepreneurial behavior: employment or unemployment, etc.) is adopted, resulting in different profit and loss values *w*, the probability of realization is *q*. Decision-makers choose entrepreneurial behavior *a* over nonentrepreneurial behavior *b* mainly based on the following basis as

(20) $$\begin{array}{c} \sum g\left(p\right)v\left(∆w-c\right)>\sum g\left(q\right)v\left(∆w-c\right). \end{array}$$

In Formula (20), ∆*w* represents the deviation of profit and loss caused by the implementation of the behavior.

### 2.3. Green Entrepreneurship Questionnaire Design

The research objects were college graduates, and a total of 507 questionnaires were distributed. Among them, 307 questionnaires were collected, and 200 paper questionnaires were distributed on the spot. Excluding the questionnaires with missing answers and inaccurate filling (the normal filling time of the questionnaire was 2.5-3.5 minutes, excluding the questionnaire star and the answer sheet with the paper questionnaire filling time less than 2 minutes), a total of 461 valid questionnaires were recovered, and the effective rate of the questionnaire was 90.9%.

#### 2.3.1. Preresearch

The survey data of this study were obtained by two methods: network distribution and field research. In order to ensure the credibility and authenticity of the questionnaire, this study will conduct on-site interviews in classrooms, libraries, study rooms, and other places and distribute the questionnaires. For network, first, the questionnaires were formed on the Questionnaire Star platform, and then the questionnaires were distributed through QQ and WeChat platforms. For field, questionnaires were distributed to major colleges and universities in the city. The conclusion of this study was drawn through the data entry, arrangement, and necessary analysis of the questionnaire. The design process of the questionnaire for this study is as follows:

Firstly, the measurement of each variable referred to mature scales that have been used many times in existing studies. Usually, the scales that have been tested by many studies have good reliability and validity, which can not only effectively shorten the time for researchers to conduct questionnaire tests, but also ensure the reliability of research results.

Secondly, since the scales referred to are mostly mature scales, literal translation and back-translation of the scales were carried out to ensure the accuracy of the content of the translated version. In order to adapt to the habit of the Chinese context, appropriate adjustments have been made to the words and expressions of the items. Before the formal investigation, this study conducted a small-scale pretest with students around the school as subjects. The pretest subjects were mainly postgraduate students around them, and the questionnaires were distributed online and on-site. 50 questionnaires were distributed, and a total of 48 were returned. Excluding the 5 invalid questionnaires with missing answers, regular answers, and not serious filling (the basis for judgment is that the filling time was less than 2 minutes), the number of valid questionnaires was 43, and the effective rate of the questionnaires was 89.6%. Reliability analysis and exploratory factor analysis were carried out on the preinvestigation data, and the Cronbach's coefficient of each variable's reliability index was greater than 0.7. The validity index KMO (Kaiser-Meyer-Olkin) value and Bartley's sphericity test results met the requirements, and the principal component analysis results showed that the variable dimension was consistent with the research design. In addition, according to the analysis results of the questionnaire data and the feedback of the survey respondents, teachers and doctoral students in the professional field were invited to discuss and evaluate. Considering that too many items in the questionnaire would affect the answering experience of the respondents, the questions about the subject's school and the current major in the basic information were deleted. The items that might cause ambiguity were adjusted accordingly to form the final version of the measurement questionnaire.

#### 2.3.2. Composition of the Questionnaire

The scales in the questionnaire of this study were standardized according to the Richter 5-level scale. There were 42 items in this survey questionnaire, 34 items in the core part, and 8 items in the basic information part. There were 7 research variables in the questionnaire, including risk tendency, ecological values, social responsibility, green entrepreneurship motivation (including three dimensions of fame and fortune motive, spiritual motive, responsibility motive), and green entrepreneurship willingness, with a total of 34 items.

The first part was the measurement scale of green entrepreneurial traits, with a total of 18 items. There were 5 items in risk propensity. Ecoenvironmental values referred to the 2007 WVS (World Values Survey) questionnaire on the Chinese public's ecoenvironmental values. There were 7 items in total to measure the ecological values of college graduates with four dimensions: the view of dedication to environmental protection, the view of economic-environment relationship, the view of environmental problem cognition, and the environmental satisfaction. The sense of social responsibility measured the sense of social responsibility from the four dimensions of social morality, sense of urgency, self-discipline, and dedication.

The second part was the green entrepreneurship motivation scale. Green entrepreneurial motivation referred to the research on entrepreneurial motivation of college graduates. The motivation of green entrepreneurship is divided into three dimensions: fame and fortune, spirit, and responsibility. Considering that this paper studies the green entrepreneurship willingness of college graduates, the question of contributing to the construction of the ecological environment was added to the responsibility motivation, with a total of 11 questions.

The third part is the green entrepreneurship willingness scale. Green entrepreneurial willingness drew on the entrepreneurial willingness measurement scale and made appropriate modifications according to green entrepreneurial willingness, with a total of 5 items. In addition, referring to previous studies by scholars, this paper selected the gender, age, educational background, whether they have received entrepreneurship education, whether they have entrepreneurial experience, whether they have work experience, whether their family members have business experience, and whether they are an only child as eight items of background information to investigate the basic information base of the tested object.

## 3. Results of Entrepreneurial Intention, Practice, and Management Path

Before the confirmatory factor analysis of the ecological value scale, the KMO and Bartlett sphericity test values were tested by SPSS25 software. The test results are shown in Table 1. It can be seen that the KMO test value of the ecological value scale was 0.922, which was greater than 0.70. The results indicated that the ecological value scale is suitable for the next factor analysis.

Confirmatory factor analysis was performed on the ecological value scale by AMOS24 software. The value of *X*^2^/dF was 0.544, which was less than 3. The values of NFI, CFI, and GFI were all greater than 0.9 and very close to 1. The value of RSMEA was less than 0.05. The above five indicators all met the requirements, indicating that the fitting degree of the ecological value model meets the requirements. The confirmatory factor fitting indicators of ecological values are shown in Table 2. Amos 24.0 is a full-featured structural equation modeling (SEM) software.

It can be seen from Table 3 that the standardized factor loadings of the seven items of ecological values are all greater than 0.5, indicating that the next step of CR and AVE tests is suitable. The calculated CR value was 0.840 (>0.7), and the AVE value was 0.568 (>0.5). The above indicators showed that the combined reliability and convergent validity of the ecological values scale are ideal. The convergent validity test of the ecological values questionnaire is shown in Table 3. CR is a reliability standard, which means that the indicators in the evaluation index system are interrelated and consistent, and there is no conflict or irrelevance. The evaluation index system is highly consistent with the performance dimension and distribution of the evaluation object.

Since each software has its own advantages and disadvantages, in order to ensure the quality of the research, multiple software verifications are carried out. Before the confirmatory factor analysis of the green entrepreneurship motivation scale, the KMO and Bartlett sphericity test values were tested by SPSS25 software. The results are shown in Table 4. KMO test value of the green entrepreneurial motivation scale was 0.880, which was greater than 0.70. Approximate chi-square value was 2088.214, and the significance probability was 0.000 (*P* < 0.001), all of which met the requirements.

It can be seen from Table 5 that the value of *X*^2^/dF was 0.2011, which was less than 3. The value of NFI was 0.733. The value of CFI was 0.820. The value of GFI was greater than 0.9 and very close to 1, and the value of RSMEA was less than 0.05. It can be judged that the fitting degree of the green entrepreneurial motivation model is acceptable. The index factors of green entrepreneurial motivation are shown in Table 5.

The standardized factor loadings of the 11 items of green entrepreneurial motivation were all greater than 0.5, indicating that the next step is suitable for the test of CR and AVE (CR is shown in Figure 3(a)). The calculated CR values of fame and fortune motive, spiritual motive, and responsibility motive were 0.869, 0.806, and 0.736, respectively, which were all greater than 0.7, and the AVE value of each variable was greater than 0.5. The above indicators showed that the combined reliability and convergent validity of fame and fortune motives, spiritual motives, and responsibility motives are very ideal (AVE is shown in Figure 3(b)).

The convergent validity test results of the green entrepreneurship intention questionnaire are shown in Figure 4. The standardized factor loadings of the five items of green entrepreneurial intention were all greater than 0.5, indicating that it is suitable for the next test of CR and AVE. The calculated CR value was 0.903 (>0.7). AVE was 0.653 (>0.5) (the results of those who were very interested in green entrepreneurship, with serious consideration about green entrepreneurship, and would like to try their best to start their own green business are shown in Figure 4(a)). The above indicators showed that the combined reliability and convergent validity of green entrepreneurship intentions were very ideal. In addition, the AVE value was also used to test the discriminant validity of the scale. The square root of the mean and the correlation coefficient between the variables are compared. The discriminant validity of the scale is good if the square root of the mean of the latent variable is greater than its correlation coefficient with other latent variables in the model (the results of those who were preparing for green entrepreneurship in the future and firmly believed that green enterprises would be established in the future are shown in Figure 4(b)). The comparison showed that the square root of the AVE value of each latent variable was larger than the Pearson correlation coefficient of this latent variable and other latent variables, so it can be proved that each variable scale has good discriminant validity.

From the statistical analysis results shown in Figure 3, it can be seen that among the respondents, males accounted for 46.9% and females accounted for 53.1%. The gender ratio of the sample was basically the same (the gender ratio is shown in Figure 5(a)). In terms of age, the proportion of the sample size was 87.9% for people aged 19-25 and 7.8% for people aged 26-30. This age distribution was in line with the age distribution of college students in all grades. The above two data showed that this survey met the requirements of random sample sampling (the proportion of age is shown in Figure 5(b)). It can also be seen from the table that in terms of educational background, the majority of the surveyed groups were college graduates. In addition, the number of people who have received entrepreneurship education only accounted for 32.2% of the total number of respondents, which showed that the current investment in entrepreneurship education in colleges is not large enough, and students' interest in entrepreneurship education also needs to be improved. The number of people with entrepreneurial experience only accounted for 11.9% of the total number of surveys, indicating that the current entrepreneurial atmosphere of college graduates is not strong enough, and the corresponding publicity and encouragement policies are not familiar to the majority of students. Meanwhile, the entrepreneurial awareness of college graduates also needs to be improved.

According to the research content of the survey report on ecological cognition, it is concluded that the ecological awareness of current college graduates is not strengthened enough. Although college graduates have a certain ecological knowledge base, their knowledge is relatively shallow, and their understanding of professional knowledge about ecological environment and relevant national policies and regulations needs to be further improved. There are differences in the mastery of different types of environmental knowledge among college graduates. Specifically, first, in terms of ecological scientific knowledge, the mastery of air quality knowledge was 66.3%, and the mastery of water environment quality was 38.7%. This shows that college students' mastery of ecological science knowledge is not comprehensive enough, and there are major problems (air quality and water environment quality are shown in Figure 6(a)). In terms of daily scientific knowledge and value awareness of environmental protection and resource conservation, there is also a phenomenon that ecological awareness is not strengthened enough (daily behavioral skills knowledge and common scientific knowledge are shown in Figure 6(b)). The mastery of daily behavior skills accounted for 85.5%, and the supervision and reporting accounted for 14.5%.

The survey on purchasing green products is shown in Figure 7. Nearly 90% of the respondents believed that it is important to purchase green food that meets the standards and green products with low pollution when shopping. But only 29.3% and 38.5% of the respondents made frequent purchases. Among them, the 18-30-year-old group was the smallest among all age groups.

The survey on working hours is shown in Figure 8. 29.91% of the respondents worked for less than one year, 19.63% for 1-2 years, 27.10% for 2-3 years, 17.29% for 3-4 years, and 6.07% for more than 4 years. The distribution of college student entrepreneur time is relatively even. With the passage of time, college student entrepreneurs may withdraw from entrepreneurship due to lack of funds, excessive pressure, project failure, social situation, and other reasons. There are relatively few people who can reach more than 3-4 years, and the others are mainly college students who have not yet encountered many pressures or have not worked for a long time.

The survey on the field of the enterprise is shown in Figure 9. The primary industry accounted for 7.94%. The secondary industry accounted for 18.23%. The tertiary industry accounted for 73.83%. College students have advanced thinking and can quickly accept new things. They themselves have some scientific and cultural knowledge, mainly involved in the field of scientific and technological services. Some of them also start businesses in agriculture and industry for their own reasons. However, there are many more college students and entrepreneurs in the service field.

There is no significant difference in the performance of students' gender, age, education, and major in green entrepreneurship willingness, indicating that different gender, age, educational level, and professional background will not have a significant impact on college students' green entrepreneurship willingness. This is different from the previous research results. The reason for this result may be because of the unique attributes of green entrepreneurial willingness, which is different from the traditional entrepreneurial willingness. But it is worth noting that when exploring the influence of family's entrepreneurial background on college students' green entrepreneurial willingness, the average score of families with entrepreneurial experience was 4.0526, and the average score of families without entrepreneurial experience was 3.6463. Significance was presented at the 0.001 level greater than 0.05. The same results as previous scholars have appeared, that is, students with entrepreneurial family background have stronger (green) entrepreneurial willingness. This may be because the students will be influenced by the family entrepreneurial atmosphere and then subtly take entrepreneurship as the main way of making a living in the future and actively think about the problems of entrepreneurship to prepare for the future. The difference analysis results are shown in Figure 10.

## 4. Conclusion

Green entrepreneurship is a way to balance ecological and commercial benefits. College graduates' green entrepreneurship is a new branch of college graduates' entrepreneurship. It has some basic characteristics and conditions that entrepreneurship should have and also has the distinctive feature of green. The connotation of sustainable development is the inexhaustible driving force for green entrepreneurship of college graduates. This study incorporates risk tendency, ecological values, and social responsibility into the evaluation of entrepreneurial intention. People with strong ecological values usually hope to practice their values through practical actions, and they can obtain a greater sense of satisfaction and achievement in the process of ecological protection. Therefore, people with strong ecological values are more likely to have the idea of green entrepreneurship out of spiritual motivations such as realizing personal value and gaining a sense of achievement. The research object selected in this study is college graduates, which has certain limitations. Although under the guidance of policy incentives and education, the main target groups of green entrepreneurship activities are college students, but there are still some green entrepreneurs who are not in school. In the future work, colleges should first focus on the education of values and sense of responsibility, guide college students to establish ecofriendly values, and cultivate their sense of social responsibility. Secondly, colleges and universities should be guided by ecological values and social responsibility to identify potential green entrepreneurs. Through publicity and guidance, a communication platform between college graduates and green entrepreneurs is built to stimulate students' green entrepreneurial motivation. In the future work, we can explore the influencing factors and guarantees of green entrepreneurship, which will make the impact of green entrepreneurship more extensive.

## Figures and Tables

**Figure 1:** Influencing factors of entrepreneurial intention.

**Figure 2:** Main techniques of the study.

**Figure 3:** Examination of green entrepreneurial motivation.

**Figure 4:** Convergent validity test results of the green entrepreneurship willingness questionnaire.

**Figure 5:** Statistics of basic information of survey respondents.

**Figure 6:** Survey content on ecological cognition.

**Figure 7:** Survey on purchasing green products.

**Figure 8:** Survey on working hours.

**Figure 9:** Aspects of the company's field survey.

**Figure 10:** Difference analysis results.

**Table 1:** KMO and Bartlett's test.

KMO sampling appropriate quantity	Related parameters	0.922
Bartlett's sphericity test	Approximate chi-square	1583.552
	df	20
	Sig	0.000

**Table 2:** Confirmatory factor fitting indicators for ecological values.

Model	Index
*X* ^2^/dF	0.544
NFI	0.997
CFI	1.134
GFI	0.997
RMSEA	0.00

**Table 3:** Convergent validity test of the ecological values questionnaire.

Variable	Item	Normalized factor loadings	Combined reliability(CR)	Average extracted variance (AVE)
Social responsibility	1. Only be a follower of social morality, but also a leader of social morality	0.745	0.840	0.568
	2. Be prepared for danger in times of peace and enhance the awareness of danger	0.767		
	3. Affect the city appearance and public environment in public places	0.681		
	4. I will actively participate in group activities	0.771		
	5. Donate after a major disaster	0.723		

**Table 4:** Green entrepreneurship motivation scale KMO and Bartlett spherical test values tested.

KMO sampling appropriate quantity	Related parameters	0.880
Bartlett's sphericity test	Approximate chi-square	2088.214
	df	54
	Sig	0.000

**Table 5:** Indicator factors of green entrepreneurial motivation.

Model	Index
*X* ^2^/dF	0.2011
NFI	0.733
CFI	0.820
GFI	0.950
RMSEA	0.49

## Data Availability

The data used to support the findings of this study are available from the corresponding author upon request.
